# Chemical characteristics of groundwater and source identification in a coastal city

This article has been retracted.

**DOI:** 10.1371/journal.pone.0256360

**Published:** 2021-08-19

**Authors:** Qun Miao, Xuefei Li, Youqin Xu, Chao Liu, Ruikang Xie, Zhihan Lv

**Affiliations:** 1 School of Environmental and Municipal Engineering, Qingdao University of Technology, Qingdao, Shandong, China; 2 Qingdao Real Estate Architectural Design Institute Co., Ltd., Qingdao, Shandong, China; 3 School of Data Science and Software Engineering, Qingdao University, Qingdao, Shandong, China; Ministry of Natural Resources North Sea Bureau, CHINA

## Abstract

A coastal city is studied in this paper. Based on 42 groundwater sampling points, a Piper diagram, the Shukarev classification, the Pearson correlation analysis, Gibbs plots and the ion proportional coefficient method are used to analyze the chemical characteristics and material source. The results show that the groundwater quality in the study area varies greatly from north to south. In the northern inland area (AREA I), the main anions and cations are $HCO_{3}^{-}$ and *Ca*^2+^, and the hydrochemical characteristics are mainly *HCO*_3_ − *Ca*, *HCO*_3_ ⋅ *SO*_4_ − *Ca* and *HCO*_3_ − *Mg*. The ion concentration distribution is uniform, and the groundwater quality is good. By using Gibbs plots and the ion proportional coefficient method, the main source of ions is the dissolution of potassium feldspar, albite and carbonate rock. In contrast, in the southern coastal area (AREA II), the main anions and cations are *Cl*^−^ and *Na*^+^, and the hydrochemical characteristics are mainly *Cl* − *Na*. The ion concentration distribution presents a strong spatial difference. The closer the groundwater sampling point is to seawater, the worse the overall groundwater quality. Evaporite dissolution, seawater intrusion, cation exchange effects and human activities are the main factors affecting the groundwater quality in this area. In conclusion, the groundwater quality in northern inland area (AREA I) is better, mainly controlled by the dissolution of rocks. The groundwater quality in southern coastal area (AREA II) changes greatly, mainly controlled by seawater.

## Introduction

With the accelerated process of global climate change, researchers have gradually realized that environmental changes and human activities have a huge impact on natural resources [1]. However, groundwater resources are easily ignored because of their strong concealment, long water quality evolution time and complex components [2]. Groundwater resources are an important part of industry and agriculture in northern China. In arid and semiarid areas, groundwater resources are not only used for industrial and agricultural development but also play an important role in ecological and environmental construction [3, 4]. Since the 1970s, owing to the steady development of the economy, water resources have been exploited on a large scale. In addition, there is the phenomenon of overexploitation and unreasonable exploitation, which directly changes the characteristics of runoff supplementation, drainage, composition and distribution. Human activities are an important consideration in the study of groundwater [5, 6].

During the processes of groundwater flow and evolution, the chemical characteristics of groundwater are mainly affected by two types of factors: natural and anthropogenic activities. First, natural factors mainly refer to the formation lithologies, geological structures and recharge conditions in the flow area. For example, because of strong rock weathering, the dissolution of rock salt and gypsum brings about the degradation of groundwater quality in the Shule River Basin. This phenomenon is less affected by human activities [7]. In addition, in the Tailai Basin [8], the supply of fissure water and karst water in the southern mountain area leads to the weathering and dissolution of silicate rocks. As a consequence, the pore water quality is affected. Moreover, the groundwater in the Marathon Basin, NE Attica, Greece, is chemically and qualitatively unsuitable for drinking purposes, whereas it is suitable for agricultural uses [9]. The groundwater quality in the coastal alluvial aquifer system is affected by several factors, such as water-rock interactions. The groundwater quality in the western coastal area of Saudi Arabia [10] is mainly affected by water-rock interactions, evaporation and seawater intrusion. Second, the anthropogenic activities factor mainly refers to the agricultural degree, industrial water discharge and groundwater exploitation. According to the study of the eastern part of Gunugsewu [11], the increasing population and various activities can add pressure to the landscapes and groundwater. Moreover, by using principal component analysis (PCA), the the karst groundwater hydrogeochemistry in the Carboniferous Taiyuan Basin have indicated that groundwater has been affected by anthropogenic activities [12]. Unreasonable human activities have caused groundwater pollution. Geochemical processes controlling the hydrochemical evolution of shallow groundwater (<200 *m*) have been studied in the Chahan Lake Basin, China [13]. Human activities (e.g., agricultural fertilizer) also significantly affect the chemical compositions, particularly $NO_{3}^{-}$ and *Cl*^−^ contents, of groundwater in recharge areas. The groundwater quality in the coastal area of the Niger Delta [14] has deteriorated due to marsh sediments and septic tank leachate caused by human activities.

In recent years, groundwater has become an important research field for many scholars, and analysis of the chemical characteristics has become the key step [15–17]. Due to the continual change in natural factors and the ceaseless influence of human activities, the source of groundwater components is more complex. The more complex the composition of groundwater, the more difficult it is to conduct research. Therefore, conducting a hydrochemical type analysis and source identification in the study area is a key task. It is extremely difficult to conduct research by using only Piper diagrams [18], principal component analysis [19], isotope tracing [20] and other methods of analyzing chemical characteristics. It is advisable to achieve new breakthroughs by integration with other fields. At present, most of the studies have realized the combination of chemical characteristic analysis and geographic information system (GIS) analysis [21, 22]. After quantitative calculation and qualitative analysis by traditional methods, GIS is used to visualize important characteristics, such as ion concentration and divisions of hydrochemical types. As a result, obscure and lengthy research results are presented in pictures. This combination greatly reduces the difficulty of applying research results to practical management.

Due to less available freshwater resources in the study area, the study area has a large amount of groundwater exploitation. Many scholars have studied the characteristics of groundwater flow, water overdraft and nitrogen pollution in drinking water in the study area. However, there are few studies on the analysis of chemical characteristics and source identification. In the Linyi Development Zone, Liu C [23] analyzed the main pollution factors and the temporal and spatial distribution of the main pollutants. In addition, based on this study, Miao S [24] applied remote sensing technology to model and invert the pollutants in the Yihe and Shuhe Rivers. In conclusion, it is very important to analyze the hydrochemical characteristics and material sources in arid areas where groundwater is extensively exploited.

Taking a coastal city as the study area, this paper analyzes the hydrochemical types by using a Piper diagram and the Shukarev classification method. Based on Pearson correlation analysis, the source of groundwater is analyzed by Gibbs plots and the ion proportional coefficient method. Finally, the concentration is visualized by images. Based on previous study results and the current groundwater situation, corresponding solutions are proposed. Eventually, this study can provide a scientific basis for the sustainable development of groundwater resources in the study area and other similar arid areas.

The rest of the paper is organized as follows: Chapter 2 introduces the related information about the study area and the data source. To illustrate the influence of location, the rest of Chapter 2 presents the groundwater system in this paper. The results and discussion about chemical characteristics and source identification are included in Chapter 3. Finally, Chapter 4 draws the conclusions.

## Materials and methods

### Study area

The study area is public. The southern part of the study area is adjacent to the sea. In addition, the study area has a continental monsoon climate and sufficient rainfall in summer, accounting for 60% of the annual precipitation. As a result, the climate can be summarized as humid and warm in summer and cold and dry in winter. The study area has undulating hills and ravines, with high terrain on both sides and low terrain in the middle. In terms of the north-south topography, the terrain is high in the north and low in the south. The geological structure of the study area is relatively simple. Magmatic rocks are the most widely distributed. The study area is rich in mineral resources. The bedrock types in this area are mainly monzonitic granite, granodiorite, gneiss, diopside and marble. According to the characteristics of the aquifer medium, the groundwater types in the study area are mostly layered rock fissure water and massive rock fissure water and a small amount of loose rock fissure water is present in the southeast.

Groundwater recharge in the study area mainly comes from atmospheric rainfall and surface water. The groundwater in the riverbed and the gently sloping sand and gravel is also laterally recharged by groundwater on both sides of the river. In addition, groundwater is discharged by evapotranspiration, radial discharge and artificial exploitation. In general, the groundwater flow direction is from north to south, which is consistent with the gradient of the terrain.

### Sample collection

From November 2013 to January 2014, 42 representative groundwater samples were collected in the study area. The location information of the study sites are shown in Table 1. The detection methods are shown in Table 2. Groundwater sampling is carried out in accordance with the operating specifications in the”Technical specificaitons for environmental monitoring of groundwater”(HJ/T 164–2020). After determining the groundwater level, well washing and stabilization parameters, use the collected water sample to clean the 500 *mL* polyethylene sampling bottle 2 to 3 times, And seal the mouth of the bottle.

**Table 1:** The geographic coordinates for the data set.

No.	Longitude	Latitude	No.	Longitude	Latitude
1	121°53′03.096″E	37°17′21.472″N	22	121°52′24.712″E	37°05′19.630″N
2	121°55′11.607″E	37°17′22.664″N	23	121°53′14.405″E	37°05′49.227″N
3	121°56′50.242″E	37°17′23.747″N	24	121°54′10.117″E	37°06′59.874″N
4	122°08′02.253″E	37°11′53.606″N	25	121°55′54.637″E	37°07′30.184″N
5	122°05′08.248″E	37°15′16.162″N	26	121°55′57.264″E	37°11′50.024″N
6	122°06′58.051″E	37°13′21.716″N	27	121°56′16.821″E	37°02′55.610″N
7	122°07′03.194″E	37°13′08.488″N	28	121°56′08.306″E	37°02′33.639″N
8	122°08′02.253″E	37°11′53.606″N	29	121°55′59.436″E	37°02′11.048″N
9	121°59′53.819″E	37°09′56.259″N	30	121°55′55.817″E	37°01′43.444″N
10	121°59′51.537″E	37°09′29.610″N	31	121°58′13.588″E	37°02′12.460″N
11	121°55′07.961″E	37°09′50.374″N	32	121°58′15.842″E	37°02′01.289″N
12	121°55′14.127″E	37°09′44.299″N	33	122°00′21.066″E	37°04′39.580″N
13	121°55′33.217″E	37°09′35.618″N	34	122°00′52.517″E	37°03′59.263″N
14	121°56′02.741″E	37°09′37.117″N	35	122°08′11.465″E	37°03′48.088″N
15	121°49′42.594″E	37°11′09.052″N	36	121°58′50.065″E	36°59′54.592″N
16	121°49′29.906″E	37°09′42.582″N	37	122°00′04.956″E	37°00′53.908″N
17	121°49′19.192″E	37°09′01.736″N	38	122°00′29.321″E	37°01′27.004″N
18	121°49′29.049″E	37°07′32.050″N	39	122°01′11.057″E	37°01′28.129″N
19	121°49′47.128″E	37°07′02.322″N	40	122°02′56.533″E	37°00′16.003″N
20	121°49′32.601″E	37°05′11.246″N	41	122°02′55.887″E	36°59′20.756″N
21	121°51′13.039″E	37°04′53.253″N	42	122°03′11.940″E	37°00′39.027″N

**Table 2:** Ion concentration detection methods and standards.

No.	Name of indicators	Standards	Detection method
1	pH	Water quality-Determination of pH value(GB 6920–86)	Glass electrode method
2	TDS	Water quality-Determination of total dissolved solids Standard examination for drinking water (GBT 5750.4–2006 8.1)	50 °*C* Drying method 180 °*C* Drying method
3	*Na* ^+^	Water quality-Determination of water cations (HJ812–2016)	Ion chromatography
4	*K* ^+^	Water quality-Determination of water cations (HJ812–2016)	Ion chromatography
5	*Mg* ^2+^	Determination of calcium, magnesium andsodium content-Flame atomic absorption spectrometry (GB/T23273.5–2009)	Flame atomic absorption spectrometry
6	*Ca* ^2+^	Determination of calcium, magnesium andsodium content-Flame atomic absorption spectrometry (GB/T23273.5–2009)	Flame atomic absorption spectrometry
7	$HCO_{3}^{-}$	Groundwater quality determination method-Titrimetric method (DZ/T0064.49–1993)	Titrimetric method
8	$SO_{4}^{2-}$	Water quality-Determination of inorganic anions ($F^{-},Cl^{-},NO_{2}^{-},Br^{-},NO_{3}^{-},PO_{4}^{3-},SO_{3}^{2-},SO_{4}^{2-}$)-Ion chromatography (HJ84–2016)	Ion chromatography
9	*Cl* ^−^	Water quality-Determination of inorganic anions ($F^{-},Cl^{-},NO_{2}^{-},Br^{-},NO_{3}^{-},PO_{4}^{3-},SO_{3}^{2-},SO_{4}^{2-}$)-Ion chromatography (HJ84–2016)	Ion chromatography

The data used in this paper comes from a cooperating unit: No.6 Institute of Geology and Mineral Resources Exploration of Shandong Province. It is a provincial public institution mainly engaged in gold exploration. As the cooperating unit of this paper, the right to use data has been authorized.

The data reliability was tested by formula 1:

$$\begin{array}{c} E=\frac{\sum m_{c}-\sum m_{a}}{\sum m_{c}+\sum m_{a}}\times 100\% \end{array}$$ (1)

where E is the relative error (%), *m*_*c*_ and *m*_*a*_ refer to the milligram equivalent concentrations (*meq* ⋅ *L*^−1^) of cations and anions in water, respectively. If the relative error was within ± 5%, the data were considered reliable. After calculation, the error of groundwater samples in the study area was less than 0.5%, indicating that all data are reliable.

### Groundwater system

Due to the particularity of the geographical location, the northern part of the study area is bordered by other cities, the southern part is coastal. In order to highlight the impact of seawater on groundwater, this paper divides the study into two areas. Based on the distance from the ocean, the study area is divided into the northern inland area (AREA I) and southern coastal area (AREA II), as is shown in Fig 1.

The data used to support the findings of this study are available from the corresponding author upon request.

**Fig 1:** Map of the study area showing the groundwater sampling sites.

## Results and discussion

### Hydrochemical types

The Shukarev classification is based on the six ion concentrations ($Na^{+},K^{+},Ca^{2+},Mg^{2+},Cl^{-},HCO_{3}^{-}+CO_{3}^{2-},\text{and}\;SO_{4}^{2-}$) in groundwater and total dissolved solids (TDS). This method combines anions and cations with a milliequivalent percentage of more than 25% in groundwater and divides it into 49 categories. Based on the percentages of the six ions’ milligram equivalent per liter, a Piper diagram is also drawn to make the water type intuitively understandable. By mapping the data in the two hydrochemical triangles in the diamond diagram, the chemical characteristics and the relative composition of groundwater can be easily explained. In this paper, we classified the data of 42 groundwater sampling sites according to the Shukarev classification method, and a Piper diagram is also drawn (Fig 2). In AREA I, the main cations were *Ca*^2+^ and *Mg*^2+^, while the main anions were $HCO_{3}^{-}$ and $SO_{4}^{2-}$. The major hydrochemical types were *HCO*_3_ − *Ca*, *HCO*_3_ ⋅ *SO*_4_ − *Ca* and *HCO*_3_ − *Mg*. In AREA II, the main cations in the groundwater were *Na*^+^, and *K*^+^, the main anion was *Cl*^−^, and the main hydrochemical type was *Cl* − *Na*. According to the results of the Shukarev classification, there were 23 groundwater hydrochemical types. The number of *HCO*_3_ hydrochemical types was the largest, accounting for 38.1% of the total samples. The *HCO*_3_ ⋅ *SO*_4_ type accounted for 26.2%, and the *Cl* type accounted for 14.3%. In summary, there were various kinds of groundwater in the study area, and its hydrochemical types differed greatly from north to south. The main types were *HCO*_3_ ⋅ *SO*_4_ − *Ca*, *HCO*_3_ − *Ca* and *Cl* − *Na*, accounting for 19.1% and 16.7% and 11.9%, respectively.

**Fig 2:** Piper diagram of groundwater points in the study area.

### Characteristics of groundwater quality indicators

Ten groundwater quality indicators, including pH, TDS, total hardness, *Na*^+^, *K*^+^, *Mg*^2+^, *Ca*^2+^, $HCO_{3}^{-}$, $SO_{4}^{2-}$ and *Cl*^−^, were screened, and their parameter characteristics were calculated and counted. In this study, we chose *mg*/*L* as the unit, except for pH, which is unitless.

In AREA I, the statistics of groundwater chemical parameters are shown in Table 3. The pH of the groundwater in this area was between 6.60 and 7.60, with an average value of 7.11. The results indicated that groundwater was weakly acidic to neutral. TDS were less than 1000 mg/L, which meant that it was freshwater. The groundwater quality met the requirements in the “Sanitary Standards for Drinking Water” (GB 5749–2006). The average was 213.36 *mg*/*L*, which was slightly hard water. The proportions of soft water (<150 *mg*/*L*), slightly hard water (150 *mg*/*L* − 300 *mg*/*L*) and hard water (300 *mg*/*L* − 450 *mg*/*L*) were 35%, 42% and 23%, respectively. All samples met the requirements of the “Sanitary Standard for Drinking Water” (GB 5749–2006) (total hardness≤450 mg/L). The order of the average values in AREA I was $HCO_{3}^{-}>SO_{4}^{2-}>Cl^{-}>Ca^{2+}>Na^{+}>Mg^{2+}>K^{+}$. Combined with the standard deviation, there was a large gap between the $HCO_{3}^{-}$ and $SO_{4}^{2-}$ averages. The coefficient of variation can eliminate the influence of the difference in the average values. When comparing the degree of dispersion among different variables, the coefficient of variation was more scientific. In AREA I, the coefficients of variation were less than 100%, which was a weak variation. The results indicated that the ion distribution was stable in AREA I.

**Table 3:** Hydrochemical indicators in AREA I.

Category	pH	*total hardness*	*TDS*	*Na* ^+^	*K* ^+^	*Mg* ^2+^	*Ca* ^2+^	$HCO_{3}^{-}$	$SO_{4}^{2-}$	*Cl* ^−^
		(*mg*/*L*)								
Maximum	7.60	380.93	721.68	72.42	8.81	44.84	107.29	198.99	188.47	117.87
Minimum	6.60	43.20	168.57	8.56	0.71	2.86	9.44	28.44	5.28	21.45
Average	7.11	213.36	378.78	35.27	1.99	22.18	48.85	100.21	78.05	52.80
Standard deviation	0.35	95.25	158.09	16.70	1.68	11.88	24.64	50.72	52.21	24.73
Coefficient of variation(%)	4.86	44.65	41.74	47.35	84.56	53.55	50.44	50.61	66.90	46.85

Table 4 shows the statistics of the chemical composition of groundwater parameters in AREA II. The pH was between 6.70 and 8.10, with an average of 7.35. This meant that the groundwater quality in this area was neutral to alkaline, while TDS was 7043.10 mg/L on average. Therefore, the groundwater was saltwater. Based on the samples in AREA II, the proportions of freshwater, brackish water and saltwater were 44%, 19%, and 37%, respectively. Only 44% of groundwater met the “Sanitary Standard for Drinking Water” (GB 5749 -2006) requirements. From the perspective of total hardness, the proportions of soft water, slightly hard water, hard water and extremely hard water were 0%, 31%, 31%, and 38%, respectively, and 62% of groundwater met the “Sanitary Standards for Drinking Water” (GB5749- 2006) requirements. The order of the average values of the ion concentration in AREA II was $HCO_{3}^{-}>SO_{4}^{2-}>Cl^{-}>Ca^{2+}>Na^{+}>Mg^{2+}>K^{+}$. Combined with the standard deviation, there was a large gap between the $HCO_{3}^{-}$. Combined with the standard deviation, some samples of *Na*^+^ and *Cl*^−^ showed a large gap between the average. The coefficients of variation of pH and $HCO_{3}^{-}$ were less than 100%, but for the other 8 indicators, they were 100%∼400%, which was a medium-strong variation. The results indicated that the above 8 indicators had a high degree of dispersion, and those ions were easily affected by the characteristics of the medium, geographic location and other factors, leading to a large concentration gap.

**Table 4:** Hydrochemical indicators in AREA II.

Category	pH	*total hardness*	*TDS*	*Na* ^+^	*K* ^+^	*Mg* ^2+^	*Ca* ^2+^	$HCO_{3}^{-}$	$SO_{4}^{2-}$	*Cl* ^−^
		(*mg*/*L*)								
Maximum	8.10	7265.21	30824.48	9872.00	374.20	1277.31	896.47	554.31	2638.58	18313.47
Minimum	6.70	172.79	255.48	16.21	0.81	27.66	22.02	71.09	48.99	35.73
Average	7.35	1829.70	7043.10	1959.38	62.49	322.28	201.41	250.51	567.03	3746.22
Standard deviation	0.35	2510.93	10758.68	3219.91	103.28	462.18	264.18	135.36	783.23	6171.60
Coefficient of variation(%)	4.71	137.23	152.75	164.33	374.20	143.41	131.16	54.03	138.13	164.74

Due to the different geographical locations, the groundwater quality in AREA I and AREA II presented significant differences. In AREA I, the main anions and cations in groundwater were $HCO_{3}^{-}$ and *Ca*^2+^, all indicators were distributed uniformly, and the groundwater quality was good. The water quality basically reached the requirements of “Sanitary Standards for Drinking Water” (GB 5749–2006). However, in AREA II, the main anions and cations were *Cl*^−^ and *Na*^+^, and the difference in the indicator distribution was more obvious. The groundwater quality in this area was poor, and most of the groundwater was saltwater and brackish water.

### Distribution characteristics of groundwater indicators

To show the distribution of groundwater components more intuitively, Spline was used in this section to expand the data in 42 detections. This method is suitable for gradually changing curved surfaces, such as ion concentration. Besides, spline has a small amount of calculation and is easy to operate. The images revealed the indicator concentration distribution in the study area (Fig 3). By combining the analysis of the indicator concentration distribution map, the results revealed that except for $HCO_{3}^{-}$, the other six ions and TDS had similar distribution patterns: low concentration in the hinterland and high concentration in the surrounding area, lower ion concentration in the north than that in the south, and lower concentration in the east than in the west. The difference in the groundwater quality in AREA I was relatively smaller. The ion concentration was uniformly distributed in this area. However, the differences between the points in AREA II were more obvious. In AREA II, the closer the point was to the sea, the higher the ion concentration and the worse the overall groundwater quality.

**Fig 3:** Images of main ion concentration distribution.

### Similarity and difference of material sources

The physical and chemical characteristics of groundwater were not only affected by various rock types but are also related to environmental factors, such as climate conditions, alternating periods of plentiful seasons and drought seasons, and geological structures [25]. Groundwater was recharged by atmospheric precipitation and rivers. After a long period of runoff, some components in the rocks penetrated the groundwater, changing the groundwater quality. In general, the evolution of the groundwater quality was affected by water-rock interactions, evaporation, interception, and diffusion.

The Pearson correlation coefficients were calculated by formula 2:

$$\begin{array}{c} \gamma =\frac{\sum_{i=1}^{n}\left(x_{i}-\bar{x}\right)\left(y_{i}-\bar{y}\right)}{\sqrt{\sum_{i=1}^{n}{\left(x_{i}-\bar{x}\right)}^{2}}+\sqrt{\sum_{i=1}^{n}{\left(y_{i}-\bar{y}\right)}^{2}}} \end{array}$$ (2)

where *γ* is the correlation coefficient. *n* is the number of samples. *x*_*i*_ and *y*_*i*_ are the the observed values of corresponding to *x* and *y*. $\bar{x}$ and $\bar{y}$ is the average of corresponding to *x* and *y*.

Groundwater quality varied greatly due to a long period of flow and was affected by various factors. With the help of Pearson correlation analysis, the correlation among different components can be clarified. First, as shown in Table 5, except for $HCO_{3}^{-}$, all 6 kinds of indicators in AREA I were significantly correlated with TDS. This result indicated that these 6 kinds of indicators were dominant factors of TDS. Second, the concentration of *Cl*^−^ was strongly correlated with *K*^+^, *Ca*^2+^ and *Mg*^2+^, revealing a similar source. It is speculated that the reason was the dissolution and evaporation of water-containing media by groundwater. This phenomenon caused precipitation of *Na*^+^ and *K*^+^ in monzonitic granite and gradual precipitation of *Ca*^2+^ and *Mg*^2+^ in marble. Third, the correlation between *Cl*^−^ and *Na*^+^, however, was low. In particular, the average *Cl*^−^/*Na*^+^ (milligram equivalent) in AREA I was 1.01, which was much lower than that in seawater (*Cl*^−^/*Na*^+^ = 1.16), indicating that *Cl*^−^ was basically not affected by seawater. Fourth, the concentrations of *Na*^+^ and *Ca*^2+^ were significantly correlated, so it can be inferred that *Na*^+^ also came from rock dissolution. Fifth, the concentration of $SO_{4}^{2-}$ was correlated with *Ca*^2+^ and *Mg*^2+^. Consequently, it can be inferred that $SO_{4}^{2-}$ came from the elution of magnesium-containing sulfate and calcium-containing sulfate in AREA I.

**Table 5:** Pearson correlation analysis of the main indicators in AREA I.

Name of indicators	*Na* ^+^	*K* ^+^	*Ca* ^2+^	*Mg* ^2+^	*Cl* ^−^	$SO_{4}^{2-}$	$HCO_{3}^{-}$	*TDS*
*Na* ^+^	1	0.311	0.556**	0.210	0.339	0.315	0.101	0.607**
*K* ^+^		1	0.745**	0.172	0.842**	0.189	-0.092	0.706**
Ca 2+			1	0.463*	0.793**	0.483*	0.139	0.884**
Mg 2+				1	0.505**	0.876**	0.357	0.666**
Cl -					1	0.479*	0.129	0.847**
$SO_{2}^{4}$						1	0.198	0.729**
$HCO_{3}^{-}$							1	0.16
TDS								1

** indicates a strong correlation at the 0.01 level (two-sided) and

* indicates a strong correlation at the 0.05 level (two-sided).

First, according to Table 6, the correlation coefficients of the main indicators were all greater than 0.7, except for $HCO_{3}^{-}$ and TDS in AREA II. The results indicated a very strong correlation among these indicators. This illustrated that these indicators were the dominant factors of TDS. Second, *Cl*^−^ had a strong correlation with *K*^+^, *Ca*^2+^, and *Mg*^2+^. It is speculated that the reason was the dissolution of calcium and magnesium rock salts, such as calcite and dolomite. Third, the concentrations of *Cl*^−^ and *Na*^+^ were also strongly correlated in AREA II, and the average *Cl*^−^/*Na*^+^ (milliequivalents) reached 1.30, which was higher than seawater. This meant that *Na*^+^ and *Cl*^−^ were affected by seawater, and seawater intrusion had already occurred. Seawater, with different types and concentrations of ions, had changed the groundwater quality. Fourth, the concentration of $SO_{4}^{2-}$ was significantly correlated with *Cl*^−^, but it showed a weak relation with *Na*^+^, which can indicate that the source of $SO_{4}^{2-}$ is more complicated. Some of the $SO_{4}^{2-}$ was brought by seawater intrusion, while others came from the dissolution of gypsum and sulfate rock. Considering that the southern coastal area was more strongly affected by human activities, the main components of potash fertilizer were *KCl* and *K*_2_ *SO*_4_. As shown in Table 6, *K*^+^ was highly correlated with *Cl*^−^ and $SO_{4}^{2-}$, and we speculated that *K*^+^, *Cl*^−^ and $SO_{4}^{2-}$ in groundwater may be affected by the use of chemical fertilizers in agricultural areas.

**Table 6:** Pearson correlation analysis of the main indicators in AREA II.

Name of indicators	*Na* ^+^	*K* ^+^	*Ca* ^2+^	*Mg* ^2+^	*Cl* ^−^	$SO_{4}^{2-}$	$HCO_{3}^{-}$	*TDS*
*Na* ^+^	1	0.947**	0.672**	0.921**	0.942**	0.578*	0.126	0.932**
*K* ^+^		1	.804**	0.968**	0.998**	0.721**	0.136	0.994**
Ca 2+			1	0.896**	0.834**	0.969**	0.263	0.860**
Mg 2+				1	0.981**	0.828**	0.183	0.986**
Cl -					1	0.753**	0.138	0.999**
$SO_{2}^{4}$						1	0.368	0.787**
$HCO_{3}^{-}$							1	0.168
TDS								1

** indicates a strong correlation at the 0.01 level (two-sided) and

* indicates a strong correlation at the 0.05 level (two-sided).

In summary, comparing the results of the Pearson correlation analysis in AREA I and AREA II, the location of the samples had affected the water quality. In AREA I, most indicators came from the dissolution of rock but were barely affected by seawater. In AREA II, some ion concentrations had been affected by seawater intrusion and human activities but hardly affected by water rock dissolution.

### Gibbs plots

In 1970, Gibbs designed a semilogarithmic coordinate system to clarify the factors affecting surface water [26]. The coordinate system set TDS as the ordinate and *Na*^+^/(*Na*^+^+*Ca*^2+^) or $Cl^{-}/(Cl^{-}+HCO_{3}^{-}$) as the abscissa. By comparing the sample water with rain, river and seawater, Gibbs summarized the factors into evaporation, rock weathering and atmospheric precipitation. Although the Gibbs plots originated in the field of surface water research, they have also been widely used in groundwater quality research [27, 28]. In the study area, the range of TDS was 168.57–30824.48 *mg*/*L*. The ratio of c(*Na*^+^)/c(*Na*^+^+*Ca*^2+^) was 0.24∼0.98, and the ratio of $\text{c}(Cl^{-})/\text{c}(Cl^{-}+HCO_{3}^{-}$) was 0.13∼0.99. According to Fig 4, most of the samples in the study area were distributed in the rock weathering-evaporative crystallization area. This result indicated that the groundwater quality was mainly affected by rock weathering. In addition, some of the groundwater quality was similar to seawater, indicating that the groundwater quality had been affected by seawater. There were also some points outside the Gibbs plots, which may be due to human activities or strong cation exchange.

**Fig 4:** Gibbs plots of the study area.

### The impact of chemical reactions on groundwater quality

By calculating the ratio of certain anions and cations, it was possible to infer the underlying lithology through which the relevant ions flow. In addition, we revealed the degree of evaporation, dissolution and water-rock interaction to study the characteristics and variation pattern of groundwater components. First, the the dissolution of rock salt was not the major factor in AREA I, some of *Cl*^−^ were also come from the dissolution of other rock. While in AREA II, seawater had affected the groundwater quality. Second, sulfate or silicate dissolution reaction rose $HCO_{3}^{-}$ and $SO_{4}^{2-}$ concentration. Third, the dissolution of evaporite was far stronger than that of carbonate rocks, especially in the AREA II. Forth, the cation exchange effect was weak in AREA I. While in AREA II, the groundwater quality was strongly affected by cation exchange.

1. *γ*(*Na*^+^) ∼ *γ*(*Cl*^−^)
  The value of *γ*(*Na*^+^) ∼ *γ*(*Cl*^−^) can reflect the source of *Na*^+^ and *Cl*^−^ in groundwater. During groundwater evolution, *Cl*^−^ does not participate in the dissolution process of water and rocks and is hardly absorbed by plants. The concentration change is only affected by evaporation. The major source of *Na*^+^ and *Cl*^−^ is rock salt dissolution.
  As shown in Fig 5(a), all the points in this study area were distributed near the 1:1 straight line, indicating that most of the *Cl*^−^ in the groundwater came from the dissolution of rock salt. In AREA I, most points were located above the 1:1 straight line. Therefore, it can be inferred that *Na*^+^ not only comes from the dissolution of rock salt but may also come from the dissolution of other sodium-containing minerals and potassium-containing minerals, such as potash feldspar and albite. In contrast, in AREA II, most points were located below the 1:1 straight line, which means *Na*^+^ is lower than *Cl*^−^. However, *Na*^+^ and *Cl*^−^ concentrations in AREA II were still much higher than those in AREA I, indicating that the concentrations had increased sharply to different extents. When the Cl- concentration was high, the *Na*^+^ concentration deviated to a greater degree. This indicated that rock salt dissolution did not completely determine the groundwater quality in AREA II. It is speculated that the groundwater quality in AREA II had been affected by seawater, which had greater concentrations of *Na*^+^ and *Cl*^−^. The concentration of *Cl*^−^ was higher than that of *Na*^+^, leading to changes in the groundwater quality in AREA II.
2.
$\gamma \left(Ca^{2+}+Mg^{2+}\right)∼\gamma \left(HCO_{3}^{-}+SO_{4}^{2-}\right)$

  The ratio of *γ*(*Ca*^2+^ + *Mg*^2+^) and $\gamma (HCO_{3}^{-}+SO_{4}^{2-})$ was usually used to infer the source of *Ca*^2+^ and *Mg*^2+^. *Ca*^2+^ and *Mg*^2+^ mainly came from the dissolution of carbonate and silicate, including minerals and rocks such as calcite and dolomite. The dissolution reaction formula of carbonate rock was as follows:
  $$\begin{array}{c} CaCO_{3}+2H_{2}CO_{3}⇌Ca^{2+}+2HCO_{3}^{-} \end{array}$$
  $$\begin{array}{c} 3CaCO_{3}+H_{2}CO_{3}+H_{2}SO_{4}⇌3Ca^{2+}+3HCO_{3}^{-}+SO_{4}^{2-} \end{array}$$
  $$\begin{array}{c} 2CaMg{\left(CO_{3}\right)}_{2}+2H_{2}CO_{3}+H_{2}SO_{4}⇌2Ca^{2+}+2Mg^{2+}+6HCO_{3}^{-}+SO_{4}^{2-} \end{array}$$
  As shown in Fig 5(b), some points were located below the 1:1 straight line, indicating that concentrations of $HCO_{3}^{-}$ and $SO_{4}^{2-}$ cannot reach the existing ion concentration merely relying on the weathering process. Therefore, sulfate or silicate dissolution also mattered.
3.
$\gamma \left(SO_{4}^{2-}+Cl^{-}\right)∼\gamma \left(HCO_{3}^{-}\right)$

  In the closed state of bays and arid areas, evaporite was a chemical sedimentary rock formed by continuous evaporation of brine. Its main components were chloride, sulfate, nitrate and borate. According to the composition, it can be divided into gypsum (*CaSO*_4_ ⋅ 2*H*_2_ *O*), anhydrite and rock salt. Carbonatite was mainly composed of carbonate minerals, such as dolomite (*CaMg*(*CO*_3_)_2_), calcite (*CaCO*_3_), and iron dolomite (*Ca*(*Fe*, *Mg*, *Mn*)(*CO*_3_)_2_). The ratio of $\gamma (SO_{4}^{2-}+Cl^{-})$ and $\gamma (HCO_{3}^{-})$ can reflect which dissolution was stronger: evaporite or carbonate rock. $\gamma (SO_{4}^{2-}+Cl^{-})$ represented the dissolution of evaporite, and $\gamma (HCO_{3}^{-})$ represented the dissolution of carbonate rock.
  According to Fig 5(c), it can be concluded that most sample points were located above the 1:1 straight line in the study area. Therefore, the dissolution of evaporite was far stronger than that of carbonate rocks. Especially in the AREA II data, the value of $\gamma (SO_{4}^{2-}+Cl^{-})$ was tens of times higher than that of $\gamma (HCO_{3}^{-})$. Compared with the AREA I data, the wide distribution of evaporites strengthened the dissolution effect, leading to changes in the groundwater composition.
4.
$\left(\gamma \left(Ca^{2+}+Mg^{2+}\right)-\gamma \left(SO_{4}^{2-}+HCO_{3}^{-}\right)\right)∼\gamma \left(Na^{+}-Cl^{-}\right)$

  Groundwater quality is affected not only by the interaction of water and rock but also by cation exchange. *Na*−*Ca* exchange is the most common cation exchange. Because the replacement capacity of *Ca*^2+^ is greater than that of *Na*^+^, the *Ca*^2+^ in the solid replaces the *Na*^+^ in the water. The reaction is as follows:
  $$\begin{array}{c} 2Na^{+}+Ca=Ca^{2+}+2Na \end{array}$$ (6)
  The magnitude of the slope of $\left(\gamma \left(Ca^{2+}+Mg^{2+}\right)-\gamma \left(SO_{4}^{2-}+HCO_{3}^{-}\right)\right)∼\gamma \left(Na^{+}-Cl^{-}\right)$ characterizes the degree of cation exchange. The main source of *Na*^+^ was the dissolution of rock salt and plagioclase, while *Cl*^−^ was mainly from the dissolution of rock salt. Therefore, *γ*(*Na*^+^ − *Cl*^−^) represented the *Na*^+^ obtained in the groundwater (except that produced by the dissolution of rock salt). The main source of *Ca*^2+^ and *Mg*^2+^ was the dissolution of rocks such as rock salt, gypsum and dolomite. $SO_{4}^{2-}$ and $HCO_{3}^{-}$ characterized the degree of dissolution of gypsum, dolomite, and calcite. Therefore,$\gamma \left(Ca^{2+}+Mg^{2+}\right)-\gamma \left(SO_{4}^{2-}+HCO_{3}^{-}\right)$ represented the extra *Ca*^2+^ and *Mg*^2+^ that was not obtained from the dissolution of gypsum, dolomite and calcite. If cation exchange was strong, the slope of $\left(\gamma \left(Ca^{2+}+Mg^{2+}\right)-\gamma \left(SO_{4}^{2-}+HCO_{3}^{-}\right)\right)∼\gamma \left(Na^{+}-Cl^{-}\right)$ should be close to -1. That was, as the *Ca*^2+^ and *Mg*^2+^ concentrations increased, cation exchange strengthened. More *Na*^+^ in the rock and soil participated in the exchange, and *γ*(*Na*^+^ − *Cl*^−^) decreased accordingly. According to Fig 5(d), the slope of the fitted straight line in AREA I was almost 0, indicating that the cation exchange effect was weak, while the slope in AREA II was close to -1, which meant that the groundwater quality in AREA II was strongly affected by cation exchange.
  Analysis concerning $\left(\gamma \left(Ca^{2+}+Mg^{2+}\right)-\gamma \left(SO_{4}^{2-}+HCO_{3}^{-}\right)\right)∼\gamma \left(Na^{+}-Cl^{-}\right)$ could supplement the conclusions obtained in the Gibbs plots. In the Gibbs plots, there were some points beyond the model. We speculated that the reason may be human interference or cation exchange interference. According to the analysis of Fig 5(d), cation exchange was relatively weak in AREA I and strong in AREA II. Therefore, it can be inferred that points beyond the Gibbs plots in AREA I were mainly affected by human activities, while they were mainly affected by cation exchange in AREA II.

**Fig 5:** Ion proportional coefficient diagrams of the study area.

## Conclusions

1. There are many hydrochemical types in the study area, and the groundwater quality differs greatly from north to south. The main anions and cations in AREA I are $HCO_{3}^{-}$ and *Ca*^2+^, and the hydrochemical types are *HCO*_3_ − *Ca*, *HCO*_3_ ⋅ *SO*_4_ − *Ca* and *HCO*_3_ − *Mg*, these three hydrochemical types account for 20.8% of the study area. The main anions and cations in AREA II are *Cl*^−^ and *Na*^+^, and the main hydrochemical type is *Cl* − *Na*, this hydrochemical type account for 8.4% of the study area.
2. The ion distribution in AREA I is uniform, while the spatial differences of *K*^+^, *Na*^+^, *Cl*^−^ and *Mg*^2+^ in AREA II are greatly affected by the environment. Ion distributions are similar, except for $HCO_{3}^{-}$. The trend decreases from inland to coastal areas. Overall, the closer to the sea, the worse the groundwater quality is.
3. Gibbs plots show that the groundwater quality in the study area is mainly affected by the weathering of rocks. Some of the sample in AREA II is extremely similar to seawater components, indicating that the groundwater quality has been affected by seawater.
4. The results of the Pearson correlation analysis method and ion proportional coefficient method show that the composition of groundwater in the study area is affected by the dissolution of rocks, seawater intrusion and human activities. The main ruling factors in AREA I are the dissolution of potash feldspar, albite and carbonate rock. Transitioning from inland to coastal areas, the groundwater quality in AREA II is also affected by seawater intrusion. The dissolution of evaporites, human activities and strong cation exchange all affect the evolution of the groundwater quality.

## Supporting information

S1 Data We upload the minimal data set as a supporting information file. It named as Data.
(CSV)
